The article "LncRNA NRON alleviates atrial fibrosis through suppression of M1 macrophages activated by atrial myocytes" was published in 2019. Journal: Biosci Rep.

# LncRNA NRON alleviates atrial fibrosis through suppression of M1 macrophages activated by atrial myocytes

**DOI:** 10.1042/BSR20192215

**Published:** 2019-11-22

**Authors:** Fei Sun, Zhixiang Guo, Chengxin Zhang, Hong Che, Wenhui Gong, Zhiming Shen, Yinglu Shi, Shenglin Ge

**Affiliations:** Department of Cardiovascular Surgery, First Affiliated Hospital of Anhui Medical University, No.218 Ji-Xi Road, Hefei 230022, China

**Keywords:** atrial fibrillation (AF), IL-12, M1 macrophages, NRON

## Abstract

The aim of the present study was to explore the role of long non-coding RNA (lncRNA) non-coding repressor of NFAT (NRON) in the atrial fibrosis and to explore whether its underlying mechanism was associated with macrophage polarization. Enzyme-linked immunosorbent assay (ELISA) analysis of pro-inflammatory cytokines revealed that NRON overexpression suppressed, whereas NRON silencing facilitated the angiotensin II (Ang II)-induced inflammatory response in primary cultured atrial myocytes. The chromatin immunoprecipitation (ChIP) results showed that nuclear factor of activated T cell 3 (NFATc3) was recruited to the promoter region of interleukin (IL) 12 (IL-12) in atrial myocytes. Further data showed that NRON overexpression suppressed, whereas NRON silencing further promoted the Ang II-induced NFATc3 nuclear transport and IL-12 expression in atrial myocytes. Moreover, RAW264.7 macrophages were incubated with the conditioned medium from the Ang II-treated atrial myocytes transfected with NRON and IL-12 overexpression vectors. IL-12 overexpression abrogated the NRON overexpression-mediated inhibition of RAW264.7 macrophage polarization to the M1-like phenotype. Additionally, mouse atrial fibroblasts were incubated with the culture medium from RAW264.7 macrophages treated as described above. IL-12 overexpression rescued the NRON overexpression-inhibited protein levels of fibrosis markers Collagen I/III in mouse atrial fibroblasts. Collectively, our data indicate that lncRNA NRON alleviates atrial fibrosis through suppression of M1 macrophages activated by atrial myocytes.

## Introduction

Atrial fibrillation (AF) is one of the most common arrhythmia of clinical significance [1], which is associated with increased morbidity and mortality [2]. The mechanisms of AF are incompletely understood. However, there have been no effective means of prevention till now. Therefore, there is greater need to identify novel therapeutic targets by deciphering the critical molecular mechanisms regulating AF.

Accumulating studies demonstrate that there are a large number of pro-inflammatory cells, such as macrophages, in the heart tissues during the development of myocardial fibrosis [3]. Once the infiltrating macrophages were activated, they could secrete various pro-inflammatory chemokines, resulting in myocardial fibrosis through interacting with cardiomyocytes or fibroblasts [4]. Macrophages are important medullary natural immune cells, the functional phenotype of macrophage can polarize into two different states (M1 and M2 macrophages) to participate in different functional immune reaction process under different local microenvironments [5]. Mounting evidence shows that after acute injury, M1-type macrophages first infiltrate into the damaged site to promote the clearance of necrotic debris, and then M2-type macrophages promote tissue healing [6]. Studies have confirmed that inhibition of macrophage M1 and promotion of macrophage M2 polarization can reduce myocardial remodeling and improve cardiac function [7,8].

Long non-coding RNAs (lncRNAs) are a subgroup of RNA transcripts greater than 200 nucleotides in length with little or no protein-coding potential [9]. LncRNAs are emerging as important regulators for various biological events through chromatin modification, as well as via transcriptional and post-transcriptional processes [11]. Nuclear factor of activated T cells (NFAT) is a remarkably sensitive transcription factor that was first identified in nuclear extracts from activated T cells. NFAT plays a critical role in the development of the heart and vasculature, musculature and nervous tissue [12]. LncRNA non-coding repressor of NFAT (NRON) was reported to function as an NFAT repressor through the inhibition of NFAT activity by reducing NFAT nuclear translocation [13]. Our previous study showed that NRON alleviated atrial fibrosis via promoting phosphorylation of nuclear factor of activated T cells 3 (NFATc3) and inhibiting its nuclear import.

The activation of macrophages is regulated by cardiac myocytes in heart diseases [14–16]. With disease condition, the inflammatory response induced by myocardial apoptosis can activate macrophages and promote myocardial fibrosis. It has been reported that NFATc3 can bind to interleukin (IL) 12 (IL-12) gene promoter in the nucleus and promote the transcription and expression of IL-12 [17]. IL-12, an inflammatory cytokine, can promote the polarization of macrophages to M1-like phenotype [18]. Hence, we hypothesized that lncRNA NRON might inhibit the transcription and expression of IL-12 in myocardial cells through inhibiting the nucleation of NFATc3, thereby regulating the interaction between myocardial cells and macrophages, regulating the macrophage M1/M2 balance and inhibiting myocardial fibrosis.

## Materials and methods

### Primary atrial myocytes culture and transfection

The mouse primary atrial myocytes were purchased from the Shanghai Institute of Cell Biology (Shanghai, China). Cells were cultured in Dulbecco’s modified Eagle’s medium (DMEM, Gibco BRL, Rockville, MD, U.S.A.) supplemented with 10% fetal bovine serum (FBS, Gibco BRL) and penicillin–streptomycin (100 IU/ml) in a humidified atmosphere of 95% air and 5% CO_2_ at 37°C.

For the cell transfection experiments, NRON overexpression vector, IL-12 overexpression vector, NRON siRNA (si-NRON) and their corresponding controls were synthesized by GenePharma Co., Ltd. (Shanghai, China). The cultured atrial myocytes were transfected with 500 ng/μl overexpression vectors and 50  nM siRNAs was performed using Lipofectamine 2000 reagent (Invitrogen, Thermo Fisher Scientific, Waltham, MA, U.S.A.) according to the manufacturer’s protocol. Finally, 48 or 72 h after transfection, transfected cells were collected and used in further experiments.

### Cell co-culture

For co-culture of atrial myocytes and macrophages, atrial myocytes were transfected with NRON and IL-12 overexpression vectors, followed by treatment with angiotensin II (Ang II) at a concentration of 1 μM. After 12 h of culture, the medium was discarded, washed twice with phosphate-buffered saline (PBS), and then the fresh medium was added and continued to cultivate. The conditioned medium was collected, filtered with a filter (Millipore, Billerica, MA, U.S.A.), and then added to RAW264.7 macrophages for 12 h of incubation.

For co-culture of macrophages and atrial fibroblasts, the culture medium from RAW264.7 macrophages treated as described above was collected and added to mouse atrial fibroblasts for 24 h of incubation.

### Quantitative real-time PCR

The mRNA expression of NRON, IL-12, inducible nitric oxide synthase (iNOS), interferon-γ (IFN-γ), arginase-1 (Arg-1), and IL-10 were detected by using quantitative real-time PCR (qRT-PCR). Total RNA was extracted from cells with TRIzol reagent (Invitrogen) following the manufacturer’s protocol. Reverse transcription was carried out using the High Capacity cDNA Reverse Transcription Kit (Applied Biosystem, Foster City, CA, U.S.A.), qRT-PCR was performed by CFX96 real-time PCR detection system (Bio-Rad, Hercules, CA, U.S.A.). Data were normalized to the reference gene *GAPDH* for each cDNA sample. The primers were as follows:

NRON-F: 5′-CAAATCCAGTTGCAAGGACC-3′;

NRON-R: 5′-AGCTCAGTCCTAGGGTAGG-3′;

IL-12-F: 5′-TTGCTGGTGTCTCCACTCATG-3′;

IL-12-R: 5′-GTCACAGGTGAGGTTCACTGTTTC-3′;

iNOS-F: 5′-CGAAACGCTTCACTTCCAA-3′,

iNOS-R: 5′-TGAGCCTATATTGCTGTGGCT-3′;

IFN-γ-F: 5′-CGGCACAGTCATTGAAAGCCTA-3′,

IFN-γ-R: 5′-GTTGCTGATGGCCTGATTGTC-3′;

Arg-1-F: 5′-AACACGGCAGTGGCTTTAACC-3′,

Arg-1-R: 5′-GGTTTTCATGTGGCGCATTC-3′;

IL-10-F: 5′-CACAAAGCAGCCTTGCAGAA-3′,

IL-10-R: 5′-AGAGCAGGCAGCATAGCAGTG-3′;

GAPDH-F: 5′-GTCTTCCTGGGCAAGCAGTA-3′,

GAPDH-R: 5′-CTGGACAGAAACCCCACTTC-3′.

### Cell viability

Cells were seeded into 96-well plates at 2.5 × 10^3^ cells per well and were given different treatments, then the OD_570_ values of different treatment groups were measured using the microplate reader (Multiskan MK3, Thermo Labsystems, Finland). All experiments were performed three times.

### Enzyme-linked immunosorbent assay

Levels of cytokines including IL-1β, tumor necrosis factor-α (TNF-α) and IL-12 were measured with their commercial Enzyme-linked immunosorbent assay (ELISA) kits (R&D Systems, Minneapolis, MN, U.S.A.) according to the manufacturer’s instructions.

### Western blot

Total proteins were extracted from cells using RIPA lysis buffer (Beyotime, Shanghai, China) and quantified with the BCA kit (Beyotime). Equal volume of protein was loaded and separated with 10% sodium dodecyl sulfate/polyacrylamide gel electrophoresis gels and transferred to polyvinylidene difluoride membrane. After blocking in 5% non-fat milk for 1 h at room temperature, the membranes were incubated overnight at 4°C with corresponding primary antibodies including Collagen I (1:1000; Abcam, Cambridge, MA, U.S.A.), Collagen III (1:1000; Abcam). Subsequently, the membranes were incubated for 2 h with secondary antibodies conjugated with horseradish peroxidase at room temperature. The ECL kit (Thermo Scientific) was used to detect immunoreactive bands according to the manufacturer’s instructions.

### Immunofluorescence staining

Briefly, the atrial myocytes were washed twice with PBS, fixed with 4% polyformaldehyde for 20 min, and then treated with 0.5% Triton-100 X at room temperature for 20 min. After being blocked in 1% bovine serum albumin overnight, cells were incubated with NFATc3 antibody (1:100, Santa Cruz Biotechnology, Dallas, TX, U.S.A.) at 4°C overnight. Subsequently, cells were washed three times with PBS, and incubated with the Alexa Fluor® 488-labeled secondary antibody (green; 1:1000) at 37°C for 30 min. After washing three times with PBS, cells were stained with DAPI in the dark and observed under a laser confocal microscope.

### Chromatin immunoprecipitation assay

Chromatin immunoprecipitation (ChIP) assay was performed using ChIP Kit (Millipore) according to the manufacturer’s instructions. Briefly, atrial myocytes were cross-linked with 1% formaldehyde for 10 min at room temperature. The cross-linking was then quenched by the addition of 0.125 M glycine. The soluble chromatin was sonicated to fragment DNA by nuclear lysis buffer. The fragmented chromatin samples were aliquoted as genomic input DNA or immunoprecipitated with IL-12 (Cell Signaling Technology, Danvers, MA, U.S.A.) and IgG (Cell Signaling Technology) and incubated at 4°C overnight. Immunocomplexes, collected by a magnetic separator, were washed and eluted with ChIP elution buffer. DNA was purified on spin columns. The ChIP products and genomic input DNA were analyzed by qRT-PCR with SYBR Green PCR Master Mix (Applied Biosystem).

### Flow cytometry

Atrial myocytes were detached with 5 mM ethylenediaminetetraacetic acid (EDTA), washed, and then resuspended in PBS supplemented with 1% heat-inactivated fetal calf serum (FCS). Cells were stained with fluorochrome–conjugated human antibodies against CD16/32 and CD206, or control antibodies, and analyzed by flow cytometry using CellQuest software package (FACS Vantage-SE, BD Immunocytometry Systems, San Diego, CA, U.S.A.).

### Statistical analysis

All data were analyzed with SPSS 16.0. Data were presented as mean ± standard deviation (SD). Student’s *t* test was used to analyze differences between two groups. One-way ANOVA analysis was used to determine differences between multiple groups. *P*<0.05 was considered to be statistically significant.

## Results

### LncRNA NRON suppresses inflammatory response in Ang II-treated atrial myocytes

To investigate the effect of lncRNA NRON on Ang II-induced atrial myocyte inflammatory response, cultured primary atrial myocytes were transfected with NRON overexpression vector and si-NRON, followed by Ang II treatment. The overexpression and knockdown efficiencies of NRON were confirmed by qRT-PCR (Figure 1A,B). MTT results indicated that Ang II treatment significantly induced cell viability in primary atrial myocytes compared with the untreated group. Importantly, NRON overexpression attenuated the Ang II-induced cell viability, whereas NRON silencing further facilitated the Ang II-induced cell viability (Figure 1C). As shown in Figure 1D–F, Ang II treatment significantly increased levels of pro-inflammatory cytokines IL-1β, TNF-α and IL-12 in cell supernatant, and the effect was attenuated by NRON overexpression but enhanced by NRON silencing. These data indicated that NRON suppressed the Ang II-induced inflammatory response in cultured atrial myocytes.

**Figure 1:** NRON suppressed inflammatory response in Ang II-treated atrial myocytes NRON overexpression vector and si-NRON and their corresponding controls were transfected into primary atrial myocytes. (**A,B**) The overexpression and knockdown efficiencies of NRON in atrial myocytes. (**C**) The effect of NRON overexpression and knockdown on atrial myocyte viability after Ang II induction was determined by MTT assay. (**D**–**F**) The levels of IL-1β, TNF-α and IL-12 in cell supernatant after Ang II induction were detected by ELISA. **P<0.01 *vs.* vector, ^##^*P*<0.01 *vs.* si-Ctrl; ^$$^*P*<0.01 *vs.* control.

### LncRNA NRON suppresses NFATc3 nuclear transport and IL-12 expression in Ang II-treated atrial myocytes

Next, we conducted a ChIP assay to examine the occupancy of IL-12 at the NFATc3 locus. The results showed that NFATc3 was recruited to the promoter region of IL-12 in atrial myocytes (Figure 2A). To gain further insight into the effect of NRON on IL-12 expression and NFATc3 nuclear transport, cultured primary atrial myocytes were transfected with NRON overexpression vector and si-NRON, followed by Ang II treatment. Results from qRT-PCR assay showed that NRON overexpression suppressed, whereas NRON silencing further elevated the Ang II-induced IL-12 mRNA expression in cultured atrial myocytes (Figure 2B). As seen in Figure 3, NRON overexpression suppressed, whereas NRON silencing enhanced the Ang II-induced NFATc3 nuclear transport in atrial myocytes. Collectively, from these results, we could clearly conclude that NRON suppressed the Ang II-induced NFATc3 nuclear transport and IL-12 expression in atrial myocytes.

**Figure 2:** NRON suppressed IL-12 expression in Ang II-treated atrial myocytes (**A**) ChIP analysis of NFATc3 binding to the IL-12 promoter. (**B**) NRON overexpression vector and si-RNA and their corresponding controls were transfected into primary atrial myocytes, then Ang II was added to induce fibrosis. IL-12 mRNA level in atrial myocytes was detected by qRT-PCR. **P<0.01 *vs.* IgG; ^##^*P*<0.01 *vs.* control; ^&&^*P*<0.01 *vs.* vector; ^$$^*P*<0.01 *vs.* si-Ctrl.

**Figure 3:** NRON suppressed NFATc3 nuclear transport in Ang II-treated atrial myocytes NRON overexpression vector and si-RNA and their corresponding controls were transfected into primary atrial myocytes, then Ang II was added to induce fibrosis. NFATc3 nuclear transport in atrial myocytes was detected by immunofluorescence staining. Scale bar: 20 μm.

### LncRNA NRON inhibits macrophage polarization to the M1-like phenotype through regulating IL-12 expression

To investigate the effect of NRON on macrophage polarization *in vitro*, the cultured atrial myocytes were transfected with NRON overexpression vector and then exposed to Ang II (1 μM), after which the conditioned medium was added to RAW264.7 macrophages. M1 macrophage was characterized by expressing CD16/32, IFN-γ and iNOS. M2 macrophage was characterized by expressing CD206, IL-10 and Arg-1. The results showed that compared with untreated group, Ang II treatment induced significant elevation of iNOS and IFN-γ mRNA expression, but this effect was partially abrogated by NRON overexpression (Figure 4A). As for the mRNA expression of Arg-1 and IL-10, they were demonstrated by the nearly four- or three-fold increase in NRON group relative to vector group (Figure 4A). Flow cytometry was then performed to detect the percentage of CD16/32+ and CD206+ cell in macrophages. As shown in Figure 4B, the percentage of CD16/32+ cells was notably increased by Ang II treatment and then significantly decreased by NRON overexpression. Meanwhile, NRON overexpression significantly induced percentage of CD206+ cells compared with the vector group (Figure 4C).

**Figure 4:** LncRNA NRON inhibits macrophage polarization to the M1-like phenotype through regulating IL-12 expression (**A**–**C**) The cultured atrial myocytes were transfected with NRON overexpression vector and then exposed to Ang II (1 μM), after which the conditioned medium was added to RAW264.7 macrophages. The mRNA levels of iNOS, IFN-γ, Arg-1 and IL-10 in macrophages were detected by qRT-PCR (A), the percentages of CD16/32+ (B) and CD206+ (C) cells were analyzed by flow cytometry. (**D**–**F**) The cultured atrial myocytes were transfected with NRON overexpression vector and IL-12 overexpression vector and then exposed to Ang II (1 μM), after which the conditioned medium was added to RAW264.7 macrophages. The mRNA levels of iNOS, IFN-γ, Arg-1 and IL-10 in macrophages were detected by qRT-PCR (D), the percentages of CD16/32+ (E) and CD206+ (F) cells were analyzed by flow cytometry. **P<0.01 *vs.* control; ^#^*P*<0.05, ^##^*P*<0.01, ^$^*P*<0.05, ^$$^*P*<0.01 *vs.* vector; ^&&^*P*<0.01 *vs.* NRON.

We further co-transfected with NRON overexpression vector and IL-12 overexpression vector into atrial myocytes and then exposed to Ang II (1 μM), after which the conditioned medium was added to RAW264.7 macrophages. Data revealed that IL-12 overexpression rescued the effect of NRON overexpression on the expression of iNOS, IFN-γ, Arg-1 and IL-10 in cells (Figure 4D). Likewise, IL-12 overexpression effectively abrogated the NRON overexpression-mediated inhibition of CD16/32+ cell percentage (Figure 4E). Furthermore, the ability of NRON overexpression to induce CD206+ cell percentage was markedly compromised when IL-12 was overexpressed (Figure 4F). Taken together, these data indicated that NRON suppressed macrophage polarization to the M1-like phenotype through inhibiting IL-12 expression.

### LncRNA NRON inhibits myocardial fibrosis by regulating macrophage M1/M2 polarization

Finally, we investigated the role of NRON in regulating myocardial fibrosis by determining expression of Collagen I and Collagen III. To this end, the culture medium from RAW264.7 macrophages which were treated as described in Figure 3 was collected and added to mouse atrial fibroblasts for 24 h of incubation. Data revealed that Ang II treatment significantly elevated protein levels of Collagen I and Collagen III, but this effect was attenuated by NRON overexpression (Figure 5A). Furthermore, the ability of NRON overexpression to inhibit expression of Collagen I and Collagen III was markedly compromised when IL-12 was overexpressed (Figure 5B). These data indicated that NRON inhibited myocardial fibrosis by regulating macrophage M1/M2 polarization.

**Figure 5:** LncRNA NRON inhibits myocardial fibrosis by regulating macrophage M1/M2 polarization (**A**) The culture medium from RAW264.7 macrophages which were treated as described in Figure 4A–C was collected and added to mouse atrial fibroblasts for 24-h incubation. The protein levels of Collagen I and Collagen III in macrophages were detected by Western blot. (**B**) The culture medium from RAW264.7 macrophages which were treated as described in Figure 4D–F was collected and added to mouse atrial fibroblasts for 24-h incubation. The protein levels of Collagen I and Collagen III in macrophages were detected by Western blot. **P<0.01 *vs.* control; ^#^*P*<0.05, ^$^*P*<0.05, ^$$^*P*<0.01 *vs.* vector; ^&&^*P*<0.01 *vs.* NRON.

## Discussion

In the present work, we found that lncRNA NRON suppressed inflammatory response in Ang II-treated atrial myocytes. Mechanistic investigation demonstrated that NFATc3 was recruited to the promoter region of IL-12 in atrial myocytes and NRON inhibited macrophage polarization to the M1-like phenotype through regulating IL-12 expression. Further results indicated that NRON inhibited myocardial fibrosis by regulating macrophage M1/M2 polarization.

Cardiac fibrosis is an important pathological condition that causes ventricular stiffness, diastolic dysfunction and arrhythmia [19,20]. To date, no therapeutic strategy has been developed to specifically target fibrosis in the heart. There is growing evidence that anti-inflammatory therapy may be a promising strategy against cardiac fibrosis. Inflammation plays a central role in the progression of cardiac fibrosis [21]. It has been suggested that Ang II could lead to the activation of NF-κB signaling to promote inflammation [19,22]. In the present study, we found that Ang II-induced inflammatory response in atrial myocytes could be suppressed by lncRNA NRON, which has been shown to play crucial roles in many developmental and pathological processes [10].

NFAT is known to be a key protein in the regulation of intracellular Ca^2+^ homeostasis and gene expression as a transcription factor in the heart, and its expression and activity are highly changed in cardiac diseases [23,24]. NFAT regulates the expression of the Il12b gene, thereby controlling the levels of the bioactive heterodimers of IL-12 p70 [17]. Our data revealed that NFATc3 was recruited to the promoter region of IL-12 in atrial myocytes, and lncRNA NRON suppressed NFATc3 nuclear transport and IL-12 expression in Ang II-treated atrial myocytes.

M1 macrophages are pro-inflammatory, and they can secrete inflammatory cytokines (e.g. IL-6, IL-12, and TNF-α). It is well-known that M1 macrophages have the typical phenotype of CD16/32^high^ and IFN-γ^high^. Besides, CD206^high^ and IL-10 ^high^ are distinctive markers of M2 macrophages [25]. In the current study, we observed that IL-12-overexpressed atrial myocytes co-cultured with macrophages showed M1-like phenotype profile including iNOS ^high^, IFN-γ^high^, CD16/32^high^ and Arg-1^low^, IL-10^low^, CD206 ^low^. These findings suggested that IL-12-overexpressed atrial myocytes could be polarized to M1-like phenotype in the Ang II-induced microenvironment. Importantly, IL-12 overexpression reversed the effect of NRON overexpression on the expression of iNOS, IFN-γ, Arg-1 and IL-10 in cells, indicating that lncRNA NRON inhibits macrophage polarization to the M1-like phenotype through suppressing IL-12 expression. However, the *in vitro* results of this preliminary study require further confirmation in animal studies.

In conclusion, lncRNA NRON alleviates atrial fibrosis through suppression of M1 macrophages activated by atrial myocytes. The present study provides an important clue to help elucidate the pathogenesis of AF and implicates NRON as a potential therapeutic target for AF.

## Abbreviations

AF: atrial fibrillation
Ang II: angiotensin II
Arg-1: arginase-1
cDNA: complementary DNA
ChIP: chromatin immunoprecipitation
DAPI: 4′,6-diamidino-2-phenylindole
GAPDH: glyceraldehyde-3-phosphate dehydrogenase
IFN-γ: interferon-γ
IL: interleukin
iNOS: inducible nitric oxide synthase
lncRNA: long non-coding RNA
NFAT: nuclear factor of activated T cell
NRON: non-coding repressor of NFAT
PBS: phosphate-buffered saline
qRT-PCR: quantitative real-time PCR
TNF-α: tumor necrosis factor-α
